The article "CD8+ T Cell-Mediated Therapeutic Antitumor Effect of an Herbal Mixture Containing Ganoderma lucidum" was published in 2023. Journal: Evid Based Complement Alternat Med.

# CD8^+^ T Cell-Mediated Therapeutic Antitumor Effect of an Herbal Mixture Containing *Ganoderma lucidum*

**DOI:** 10.1155/2023/9630816

**Published:** 2023-04-28

**Authors:** Shun Takaku, Masumi Shimizu, Rimpei Morita

**Affiliations:** ^1^Department of Microbiology and Immunology, Nippon Medical School, Tokyo 113-8602, Japan; ^2^Center for Medical Education, Nippon Medical School, Tokyo 113-8602, Japan

## Abstract

Although Kampo—a traditional Japanese herbal medicine—contributes in the control of tumor growth *in vivo* in experimental animals, most of the antitumor effects are prophylactic and not therapeutic. In this study, we determined whether oral administration of an herbal mixture containing *Ganoderma lucidum* (WTMCGEP; *Wisteria floribunda*, *Trapae fructus*, *Myristica fragrans*, *Coicis semen*, *Ganoderma lucidum*, *Elfvingia applanata*, and *Punica granatum*), anecdotally used in Japan for the palliative care of patients with cancer, exhibits a therapeutic effect on tumor growth *in vivo* in a hypodermic murine CT26 colorectal tumor model. An *in vitro* tumor assay revealed that WTMCGEP extract has some direct influence over suppression of tumor growth. In wild-type BALB/c mice, WTMCGEP did not show any antitumor effect *in vivo*. However, in BALB-CD1d^−/−^ mice with partly mitigated immunosuppression by reason of them being devoid of both antitumoral type I and immunosuppressive type II natural killer T (NKT) cells, WTMCGEP therapeutically suppressed tumor growth. CD8^+^ T cell depletion significantly accelerated tumor growth in WTMCGEP mice; therefore, its antitumor activity was primarily in a CD8^+^ T cell-dependent manner. Regarding immunosuppressive cells in tumor-bearing CD1d^−/−^ mice, WTMCGEP did not influence the abundance of tumor-infiltrating CD4^+^ and Forkhead box protein 3^+^ regulatory T cells. However, it reduced both intratumoral and splenic Ly6G^+^ Ly6C^lo^ polymorphonuclear myeloid-derived suppressor cells, which were most likely involved in tumor growth inhibition related to higher frequency of intratumoral CD107a^+^ CD8^+^ T cells in these mice. Overall, these data illustrate that the deficiency of NKT cells urges WTMCGEP to exert a therapeutic antitumor effect mainly through CD8^+^ T cells. Our efforts are the first to scientifically demonstrate the WTMCGEP's contribution to tumor immunity.

## 1. Introduction

Kampo, traditional Japanese herbal medicine, is often used in patients with cancer based on the theory that it helps reduce their various complaints or adverse events associated with chemotherapies, surgical operation, and radiation therapies [1–3]. Moreover, some prescriptions show antitumor effect in several mouse tumor models [4–11], although they remain controversial. Recently, we demonstrated the antitumor effect of Juzentaihoto (JTT) (Shi-Quan-Da-Bu-Tang in Chinese and Sipjeondaebo-Tang in Korean) in CD1d^−/−^ mice whose immune-suppressing effects were partly palliated because of the loss of both antitumoral type I and immunosuppressive type II natural killer T (NKT) cells [12]. However, most reports on the antitumoral effect of Kampo, including our study, have described Kampo as a prophylactic agent, but not as a therapeutic one. In cancer, therapeutic agents are more desirable.

Apart from Kampo, natural herbs believed to have anticancer activity are quite a few. Among them, *Ganoderma lucidum* has an anticancer effect *in vitro* and *in vivo*, although it remains controversial [13–16]. In Japan, there is an herbal mixture named WTMCGEP that contains *Ganoderma lucidum* [17]. It comprises seven herbs, namely, *Wisteria floribunda*, *Trapae fructus*, *Myristica fragrans*, *Coicis semen*, *Ganoderma lucidum*, *Elfvingia applanata*, and *Punica granatum*. Besides *Ganoderma lucidum*, five remaining ingredients other than *Trapae fructus* have been reported to have some antitumoral activity [18–22]. The origin formula of WTMCGEP included *Wisteria floribunda*, *Terminalia chebulae*, *Trapa natans*, and *Coicis semen* (WTTC), which has been used for treating cancers in Japan since the 1960s [23]. Hijikata then modified WTTC to WTTCGE, a formula containing WTTC, *Ganoderma lucidum,* and *Elfvingia applanata*, and finally, developed the present form to improve its antiviral effects [17, 24, 25]. In particular, it has been reported that a formula containing WTMCGEP plus *Panax ginseng* (WTMCGEPP) suppressed herpes zoster-related pain in five Japanese patients with shingles [17]. These modified WTTC formulas have also been empirically prescribed to mitigate various complaints associated with cancers, such as ascites, general fatigue, and pain. Although almost all reports on these formulas seem to be anecdotal, these formulas are believed to be relatively safe and could be used for a long time in patients with cancer. Moreover, clinicians and pharmacists can easily access WTMCGEP as formulated powders in Japan. Therefore, investigating on a more scientific level whether WTMCGEP exerts anticancer effects in appropriate small animal models would be worthy.

In this study, in a hypodermic murine syngeneic CT26 colorectal tumor model, we evaluated the therapeutic antitumoral effect of oral administration of WTMCGEP.

## 2. Materials and Methods

### 2.1. Animals

Inbred BALB/c and BALB/c CD1d^−/−^ mice were procured from CLEA Japan (Tokyo, Japan) and Jackson Laboratory (Bar Harbor, ME, USA), respectively. The mice were categorized in groups of five and housed in filter cages, including females (>six weeks old), in all research and preserved in a temperature-restrained, specific-pathogen–free animal facility. The mice were subjected to constant 12 h light/12 h dark cycle and allowed to have water without any obstacle and *ad libitum* reach to food as indicated. The Animal Care and Use Committee at Nippon Medical School (Tokyo, Japan), which acquired the external validation from the Japanese Association for Laboratory Animal Science, approved the entire experiments (Permit No. 2020-020). All the animal experiments were appropriately conducted per the norms provided for the laboratory animals, Nippon Medical School, Act on Welfare and Management of Animals and Standards Related to the Care and Keeping and Reducing Pain of Laboratory Animals. Each experiment included 3–5 mice/group.

### 2.2. The Herbal Mixture WTMCGEP

The herbal mixture containing *Ganoderma lucidum*, named WTMCGEP, comprises seven herbs (i.e., *Wisteria floribunda*, *Trapae fructus*, *Myristica fragrans*, *Coicis semen*, *Ganoderma lucidum*, *Elfvingia applanata*, and *Punica granatum*) (Table 1). All herbs were extracted using 11-fold hot water (weight/weight) at 95°C for 2.5 h. After filtration, the filtrate was condensed through a spray drying. We purchased WTMCGEP from Tochimoto Tenkaido & Co. (Osaka, Japan) as preservative-free pure powder. Subsequently, we used a moderate-fat diet as a control (Oriental Yeast Co., Tokyo, Japan). The mice were provided with a either the control diet or the mixture of control diet and WTMCGEP (2.0%; termed as WTMCGEP diet). To obtain the herbal extract for *in vitro* use, 100 mg of powdered WTMCGEP was dissolved in 1 ml of dimethyl sulfoxide (DMSO) (Nakarai tesque, Kyoto, Japan), and this mixture was nurtured for 24 h with shaking on a water bath at 37°C. Thereafter, it was centrifuged for 30 minutes at 20°C and 13,000 rpm. At last, its supernatant was collected as a stocked WTMCGEP extract.

### 2.3. Tumor Cell Lines

The *N*-nitro-*N*-methylurethane-induced BALB/c murine colon carcinoma CT26 cell line was obtained from the American Type Culture Collection (Manassas, VA, USA) and maintained in RPMI-1640 complete medium (Thermo-Fisher Scientific, Inc., Waltham, MA, USA). Supplements of 10% fetal calf serum (FCS) (Sigma–Aldrich; Merck KGaA, Darmstadt, Germany), penicillin (100 U/mL), streptomycin (100 *μ*g/mL), L-glutamine (2 mM), sodium pyruvate (1 mM), nonessential amino acids, HEPES (10 mM), MEM vitamin solution, and 2-mercaptoethanol (5 × 10^−5^ M) were provided to the medium.

### 2.4. In Vitro Tumor Assay with WTMCGEP

CT26 cells were positioned along 96-well plates (5 × 10^3^ cells/well) and cultured for 24 h at 37°C. Following discarding the culture supernatant, stocked WTMCGEP extract for *in vitro* use was diluted with CT26 culture medium, passed through 0.22 *μ*m filters for sterilization, and then added to each well at various concentrations (2 mg/ml, 1 mg/ml, 0.5 mg/ml, 0.25 mg/ml, 0.125 mg/ml, 0.0625 mg/ml, and 0.03125 mg/ml). Since WTMCGEP extract was originally dissolved in DMSO, we also prepared a series of control wells with CT26 culture medium, including the corresponding concentration of DMSO (2%, 1%, 0.5%, 0.25%, 0.125%, 0.0625%, and 0.03125%, respectively). Following a 24 h incubation, cell viability was assessed using a Cell Counting Kit-8 (Dojindo Laboratories, Kumamoto, Japan) in lines with the maker's guidelines. Because the prepared samples were divided into three types; those without WTMCGEP nor DMSO, those with DMSO, and those with WTMCGEP + DMSO, results were calculated as the percentage of viability = (OD at 450 nm of the sample with DMSO or WTMCGEP + DMSO − OD at 450 nm of blank)/(OD at 450 nm of the sample without DMSO nor WTMCGEP − OD at 450 nm of blank) × 100.

### 2.5. In Vivo Tumor Assay and Antibody Treatment

The mice subcutaneously received 50,000 CT26 cells in 200 *μ*L cold Dulbecco's phosphate-buffered saline (DPBS) (Thermo-Fisher Scientific) on day 0 and were fed with either the control or WTMCGEP diet for twenty-eight days soon after tumor challenge. In the subgroup of the experiments, some CD1d^−/−^ mice were intraperitoneally injected with 0.2 mg of anti-CD8 mAb (clone, 2.43, cat. no.: BE0061; Bio X Cell, West Lebanon, NH, USA). The following temporal targets were considered: first and second day before tumor cell inoculation and 4^th^, 7^th^, 10^th^, and 14^th^ days following tumor cell inoculation. A caliper gage was used to measure the tumor area twice a week per this calculation; tumor length × width measured in mm. When the tumor area was <100 mm^2^ on 28^th^ day post tumor challenge, the mice were taken as “survived” [26].

### 2.6. Isolation of Tumor-Infiltrating Lymphocytes

For the isolation of tumor-infiltrating lymphocytes (TILs), tumors were sectioned from the mice and assimilated using 1 mg/mL collagenase (Roche Diagnostics GmbH, Mannheim, Germany) for forty-five minutes at temperature of 37°C. The resultant was subsequently softly creased to make the mass homogenous and sieved using a nylon filter mesh. For their purification, the collected leukocytes, via the latter process, were subsequently isolated from the polluting tumor cells using Lympholyte-M (CEDARLANE, Burlington, NC, USA) as per the maker's manual.

### 2.7. Flow Cytometric Analysis

For the determination of the expression of the cell surface molecules, flow cytometry through a FACSCanto II flow cytometer (Becton Dickinson Immunochemical Systems, Mountain View, CA) was performed. Briefly, cold DPBS (2 mL) was used to wash the isolated TILs and spleen cells, then stained using dilute Zombie NIR™ dye (BioLegend, San Diego, CA, USA) at 1:500 in DPBS at normal room temperature without light for a duration of fifteen minutes, and splashed again with DPBS with 2% heat-inactivated FCS and 0.1% sodium azide (FACS buffer). For minimizing the union of nonspecific antibody to the Fc receptors, the isolated cells were incubated with 0.5 *μ*g anti-CD16/CD32 (clone 2.4G2, cat. no.: 14-0161; eBioscience, Inc., San Diego, CA, USA) at 4°C for a duration of fifteen minutes. Following that, the pertinent antibodies were utilized to stain for half an hour at 4°C. The antibodies used were as follows: PE/Cy7-conjugated anti-CD3 (clone 17A2, cat. no.: 100220), FITC-conjugated anti-CD4 (clone GK1.5, cat. no.: 100405), FITC-conjugated anti-CD8*β* (clone YTS156.7.7, cat. no.: 126606), PE-conjugated anti-CD107a (clone 1D4B, cat. no.: 121611), PECy7-conjugated anti-CD11b (clone M1/70, cat. no.: 101215), APC-conjugated anti-CD45 (clone 30-F11, cat. no.: 103112), APC/Cy7-conjugated anti-CD45 (clone 30-F11, cat. no.: 103116), FITC-conjugated anti-Ly6G (clone 1A8, cat. no.: 127606), and PE-conjugated anti-Ly6C (clone HK1.4, cat. no.: 128007). We purchased all antibodies from Biolegend. These stained cells units were splashed once using 2 mL FACS buffer and subsequently fixed with 300 *μ*L 1x Stabilizing Fixative (BD Biosciences).

For the staining of intracellular Forkhead box protein 3 (Foxp3) to identify CD4^+^ Foxp3^+^ T cells in TILs, after surface staining using anti-CD3, -CD4, and -CD45, 2 mL cold FACS buffer was used to wash the stained cells once. Following this, the cell units were secured with 1 mL fixation/permeabilization solution (eBioscience) at a temperature of 4°C for 30 min and then cleansed two times using 2 mL 1 × permeabilization buffer (eBioscience) and stained with 0.4 *μ*g PE-conjugated anti-Foxp3 (clone FJK-16s, cat. no.: 12-5773-80; eBioscience) at 4°C for 30 min. The cells were cleansed two times using 2 mL 1 × permeabilization buffer and suspended in cold FACS buffer.

For each sample, we obtained 3000–10000 events, whose data were subsequently interpreted through FlowJo (version 9.3.1; Tree Star, Inc., Ashland, OR, USA).

### 2.8. Statistical Analysis

Following tests were used for interpreting the study outcomes: for parametric data Student's *t* test was used, nonparametric data were analyzed using Mann–Whitney *U*-test, Log-rank test, and two-way repeated measures analysis of variance (ANOVA), followed by post hoc Sidak's multiple comparisons test using Prism 6 (version 6.0 d; GraphPad Software, Inc., La Jolla, CA, USA). Differences with *p* values of <0.05 were considered statistically significant.

## 3. Results

### 3.1. WTMCGEP Extract Has a Direct Impact on the Inhibition of CT26 Tumor Growth In Vitro

To evaluate whether WTMCGEP affects tumor cell growth *in vitro*, CT26 cells were cultured *in vitro* with or without serially diluted WTMCGEP extract for 24 h. Then, their viability was assessed by Cell Counting Kit-8 (Dojindo Laboratories), as described in the “Materials and Methods” section. As shown in Figure 1, the CT26 cell life was markedly reduced in the presence of various concentrations of WTMCGEP extract (1 mg/ml, 0.5 mg/ml, and 0.25 mg/ml). These data suggest that WTMCGEP has a direct impact on the suppression of tumor growth *in vitro*.

### 3.2. WTMCGEP Therapeutically Suppresses Tumor Growth in CD1d^−/−^ Mice Mainly in a CD8^+^ T Cell-Dependent Manner

We explored if the oral administration of WTMCGEP exerts antitumor effect *in vivo*. To attain this, WT BALB/c or BALB-CD1d^−/−^ mice were hypodermically injected with 5 × 10^4^ CT26 cells. Subsequently, the mice were nourished using the control diet or WTMCGEP diet for a duration of 4 weeks. As shown in Figures 2(a) and 2(b), WTMCGEP did not influence tumor growth in the WT mice. In comparison, although we and other investigators have reported that tumors grew markedly slower in CD1d^−/−^ mice than those in WT mice [26, 27], WTMCGEP significantly accelerated tumor growth inhibition in such CD1d^−/−^ mice (Figures 2(c) and 2(d)). To elucidate whether the antitumor effect of WTMCGEP depends on CD8^+^ T cells, CD1d^−/−^ mice fed with or without the WTMCGEP diet were treated with anti-CD8 monoclonal antibodies *in vivo* before and after tumor challenge. As illustrated in Figures 2(c) and 2(d), the depletion of CD8^+^ T cells *in vivo* almost canceled the antitumor effect of WTMCGEP in the mice, although CD8-depleted mice fed the WTMCGEP diet still demonstrated a marginal but significant antitumor effect *in vivo* compared to those fed the control diet. These findings indicate that CD8^+^ T cells play pivotal roles in maximizing the therapeutic antitumor effect of WTMCGEP in CD1d^−/−^ mice.

### 3.3. WTMCGEP Augments Intratumoral CD8^+^ T Cell Activity in CD1d^−/−^ Mice

Because CD8^+^ TILs are known to back the enhancement of antitumoral immunity [28], we explored the abundance of intratumoral degranulation marker CD107a^+^ CD8^+^ T cells in CD1d^−/−^ mice nourished with a control or WTMCGEP diet 28 days after tumor challenge. As shown in Figures 3(a) and 3(b), the frequency of such TILs significantly increased in the WTMCGEP-treated mice compared to control mice. The above results convey that the elevation of CD107a^+^ CD8^+^ TILs is associated with the attenuation of tumor growth in WTMCGEP-treated mice.

### 3.4. WTMCGEP Has No Effect on the Abundance of Intratumoral CD4^+^ Foxp3^+^ Regulatory T Cells

Various immunosuppressive cells are known to dampen antitumor immunity, among which CD4^+^ regulatory T (Treg) cells are one of the hurdles for immune surveillance against cancer [29]. Prophylactic depletion of such Treg cells augmented antitumoral immunity among both WT [26, 30, 31] and CD1d^−/−^ [27] mice hypodermically injected with CT26 tumors. Moreover, a recent study has revealed that intratumoral Treg depletion by anti-CD25 immunotoxin contributes to the induction of CD8^+^ T cell-mediated systemic antitumor immunity [32]. Therefore, we evaluated the abundance of intratumoral CD4^+^ Treg cells in CD1d^−/−^ mice nourished with the control or WTMCGEP diet on day 28 after the tumor challenge. As shown in Figures 4(a) and 4(b), there was no difference in the abundance of CD4^+^ Treg cells between the two groups. These findings suggest that WTMCGEP did not affect the abundance of intratumoral Treg cells in CD1d^−/−^ mice.

### 3.5. WTMCGEP Decreases the Number of Both Intratumoral and Splenic Polymorphonuclear Myeloid-Derived Suppressor Cells in CD1d^−/−^ Mice

Besides Treg cells, myeloid-derived suppressor cells (MDSCs) are the principal immunosuppressive cells in tumor-bearing hosts [33, 34]. In practice, the major murine types of MDSCs are known as CD11b^+^ Ly6G^+^ Ly6C^lo^ polymorphonuclear MDSCs (PMN-MDSCs) and CD11b^+^ Ly6G^−^ Ly6C^hi^ monocytic MDSCs (M-MDSCs) [35]. Thus, we measured the frequency of intratumoral MDSCs in CD1d^−/−^ mice nourished with the control or WTMCGEP diet on day 28 after the tumor challenge. As shown in Figures 5(a) and 5(b), a marked reduction in intratumoral PMN-MDSCs' numbers was observed in mice nourished with the WTMCGEP diet however not in control diet. Furthermore, splenic PMN-MDSCs were also significantly reduced in WTMCGEP-treated mice (Figures 5(c) and 5(d)). In contrast, no significant differences in the proportion of M-MDSCs were observed between the control and WTMCGEP groups in neither TILs nor spleens (Figures 5(a)–5(d)). To explore if both the administration of WTMCGEP and the loss of NKT cells were necessary for the reduction of PMN-MDSCs in tumor-bearing mice, we determined the abundance of MDSCs in WTMCGEP-treated WT mice (Figures 5(e)–5(h)). As anticipated, WTMCGEP had no influence on the occurrence of PMN-MDSCs (Figures 5(e), 5(f) left, 5(g), and 5(h) left) and M-MDSCs (Figures 5(e), 5(f) right, 5(g), and 5(h) right) in these mice. As our previous study has revealed that PMN-MDSCs derived from CT26-bearing mice could function as immunosuppressive cells [12], these observations imply that the reduction of both local and systemic PMN-MDSCs plays crucial roles in the enhancement of antitumor immunity in CD1d^−/−^ mice fed with the WTMCGEP diet.

## 4. Discussion

Recently, we reported that JTT has antitumor effects on BALB-CD1d^−/−^ mice in a prophylactic setting, in which mice had been fed with a JTT-containing diet from 14 days before the CT26 tumor challenge for 42 days [12]. Based on these findings, we have sought an herbal mixture, other than JTT, to show the therapeutic antitumor effect in murine tumor models and conducted this study. *In vitro*, WTMCGEP extract had some direct antitumor effects (Figure 1). *In vivo*, we exemplified that oral administration of this herbal mixture therapeutically inhibited tumor growth in CD1d^−/−^ mice but not in immune-competent BALB/c mice (Figures 2(b) and 2(d)). Furthermore, CD8^+^ T cells were necessary for the maximization of WTMCGEP's antitumor effect (Figure 2(d)), and the frequency of CD107a^+^ CD8^+^ TILs was significantly elevated in WTMCGEP-treated mice compared to that in control mice (Figure 3). These findings emphasize the pivotal role of WTMCGEP in reinforcing antitumor immunity through CD8^+^ T cells in a tumor-bearing host on the condition that immunosuppression is partly mitigated because of deficiency of NKT cells. Although six of the seven ingredients of WTMCGEP have already been known to possess some antitumor properties [13–16, 18–22], only anecdotal evidence on the antitumor effect of this mixture itself exists. Therefore, to our best knowledge, this is the first time when WTMCGEP's contribution to enhancing the immunological antitumor effect *in vivo* is shown.

In a hypodermic CT26 tumor model, CD4^+^ Foxp3^+^ Treg cells are the predominant immunosuppressive cells. In particular, a recent study revealed that the regulation of intratumoral Treg cells enhances systemic antitumor immunity [32]. Therefore, we planned to explain whether WTMCGEP affects intratumoral CD4^+^ Treg cells in CD1d^−/−^ mice. However, this herbal mixture had no influence over the Treg cells numbers in CT26-bearing CD1d^−/−^ mice (Figure 4).

MDSCs have been regarded as a barrier to many cancer immunotherapies [36]. In our previous research, we reported that the abundance of intratumoral, but not splenic, PMN-MDSCs was significantly reduced in CT26-bearing CD1d^−/−^ mice fed the JTT diet related to the control diet [12]. Thus, we next measured the frequency of MDSCs in these mice nourished with the control or WTMCGEP diet. Distinct from JTT, the proportion of PMN-MDSCs was substantially lesser in TILs and spleens resulting from WTMCGEP mice than in those derived from control mice (Figures 5(b) left and 5(d) left). As such a reduction was not observed in tumor-bearing WT mice fed the WTMCGEP diet (Figures 5(f) left and 5(h) left), these data suggested that WTMCGEP's antitumor effect was associated with a decrease in local and systemic PMN-MDSCs in the absence of NKT cells. Recently, Wang et al. has shown that *Ganoderma lucidum* polysaccharide modulates the differentiation and inhibition of MDSCs through the CARD9-NF-kB-IDO pathway in a murine Lewis lung cancer model [37]. Although a precise mechanism is yet to be elucidated, the reduction in PMN-MDSCs in tumor-bearing WTMCGEP mice may be partially mediated by *Ganoderma lucidum*, which is one of the major components of this mixture.

Among the seven ingredients of WTMCGEP, *Ganoderma lucidum* may be the most studied as an anticancer agent and is known to have anticancer effects *in vitro* and *in vivo*, controversies remain [13–16]. However, the five remaining ingredients, other than *Trapae fructus,* have also been reported to have anticancer properties [18–22]. Therefore, WTMCGEP's antitumor effect may not depend on or may be more potent than *Ganoderma lucidum* alone.

Notably, WTMCGEP had no effect on tumor development in immunocompetent WT mice (Figure 2(b)). Moreover, compared with CD1d^−/−^ mice, tumor-bearing WT mice presented with no difference in the PMN-MDSC population in the presence or absence of WTMCGEP (Figures 5(f) left and 5(h) left). The antitumor type I NKT and immunosuppressive type II NKT cells found in WT mice functionally regulated each other. However, it is known that type II NKT cells lead type I NKT cells in tumor immunity [38]. Consequently, in several tumor models, CD1d^−/−^ mice falling short on both kinds of NKT cells showed an antitumor or antimetastatic effect at one level or another [26, 39–43]. Furthermore, IL-13 manufacture by type II NKT cells has been reported to contribute to the maintenance of CD11b^+^Gr-1^+^MDSCs via the IL-13R-STAT6 pathway in tumor-bearing mice [41, 44]. Therefore, even if WTMCGEP had some negative effects on the survival of PMN-MDSCs in tumor-bearing hosts, type II NKT cells might more strongly support the maintenance of such MDSCs. In WT mice, WTMCGEP treatment might be unable to reduce the population of PMN-MDSCs, probably due to the presence of type II NKT cells, thereby leading to failure of tumor suppression. In contrast, IL-13 inhibitor has been observed to be a pivot in the enhancement of antitumor immunity in some tumor models [39, 40, 45]. Given that IL-13 is expected to support the maintenance of MDCSs, a trial combining IL-13 blockade with oral administration of WTMCGEP for promoting effective tumor eradication in immunocompetent hosts should be considered. The effectiveness of such a combination needs to be confirmed in further studies.

Furthermore, the outstanding antitumor effect of WTMCGEP observed in CD1d^−/−^ mice suggests that combination therapy using this herbal mixture and other current cancer therapies prevents immunosuppression. Consistent with our concept, it has been reported that JTT augments the antimetastatic effect of anti-PD1 antibody against B16 mouse melanoma cells [46]. Moreover, JTT and Ninjin'yoeito (NYT; Ren-Shen-Yang-Rong-Tang in Chinese) have been described to synergize the antitumor effect in conjunction with tumor vaccines [9, 11]. Particularly, our previous study has reported that NYT may contribute to the reduction of CD4^+^ Treg cells in the spleens and tumor-draining lymph nodes derived from CT26-bearing WT BALB/c mice inoculated with irradiated tumor vaccine prophylactically [11]. As the components of these two Kampo medicines and WTMCGEP do not overlap, WTMCGEP may be an attractive option to synergize the antitumor effects in conjunction with these Kampo medicines and tumor vaccines.

However, there may be limitations in this study. First, our study about WTMCGEP was based on the results of one tumor cell line (CT26). Moreover, we were unable to check whether WTMCGEP shows antitumor effects in mouse strains such as C57/BL6 and C3H/HeN, other than BALB/c. To generalize our findings, studies are needed in the future to elucidate the *in vivo* antitumor effect of WTMCGEP against tumor cells derived from various mouse strains. Second, given that the duration of our *in vivo* tumor assay was 28 days, the long term antitumor effect of WTMCGEP could not be clarified. Third, it should be noted that WTMCGEP still possessed a marginal but significant antitumor effect *in vivo* in the absence of CD8^+^ T cells (Figures 2(c) and 2(d)). Therefore, the precise mechanism of the CD8-independent antitumor effect by WTMCGEP should be elucidated in the future. Finally, the safety of WTMCGEP should be also considered. WTMCGEP is believed to be almost free from toxicity because this mixture or its derivatives have been empirically used for more than 60 years in Japan [23] for various complaints of patients with cancer as anecdotally described as well as for palliating symptoms in various viral infections, like herpes simplex virus, varicella zoster virus, Epstein–Barr virus, and human cytomegalovirus [17, 24, 25]. Moreover, WTMCGEP-treated mice seemed to be healthy throughout our study. Nonetheless, WTMCGEP should be still consumed carefully because, for example, in *Ganoderma lucidum* alone, there are few cases of adverse effects and drug interactions reported in the literature [15]. Therefore, large-scale controlled studies will be necessary to elucidate the safety of this mixture.

## 5. Conclusions

To the best of our knowledge, it may be concluded that our study is the first to scientifically demonstrate WTMCGEP's contribution to the augmentation of CD8^+^ T cell-mediated antitumor immunity in CD1d^−/−^ mice with partly attenuated immunosuppression by reason of the deficiency of NKT cells. Although the characteristics of WTMCGEP as an anticancer agent has yet to be fully elucidated, current study sheds light on this herbal mixture as a promising and practical antitumor adjuvant.

## Figures and Tables

**Figure 1:** WTMCGEP extract has a direct impact on the suppression of CT26 tumor growth in vitro. CT26 cells were seeded in 96-well plates (5,000 cells/well) and cultured for 24 h at 37°C. After removing the culture supernatant, these cells were further incubated with WTMCGEP at the indicated concentrations for 24 h. Then, *in vitro* CT26 viability was accessed by Cell Counting Kit-8 as described in the “materials and methods” section. Data represent the means ± SEM of five independent experiments. Statistical significance between values obtained for WTMCGEP-treated (WTMCGEP) and WTMCGEP-untreated (DMSO control) wells was determined by a two-way repeated measures ANOVA, followed by a post hoc Sidak's multiple comparisons test. ^*∗∗∗*^*p*  <  0.0003, ^*∗*^*p*  <  0.03.

**Figure 2:** Oral administration of WTMCGEP therapeutically suppresses tumor growth in CD1d^−/−^ mice, mainly in a CD8^+^ T cell-dependent manner. WT BALB/c (a and b) or BALB-CD1d^−/−^ (c and d) mice were subcutaneously challenged with 5 × 10^4^ syngeneic CT26 cells. Subsequently, the mice were fed either the control or WTMCGEP diet for 4 weeks after the tumor challenge. In experiments with CD1d^−/−^ mice, we added two more groups that included control- or WTMCGEP-diet mice treated with anti-CD8 monoclonal antibody (mAb) *in vivo*. The tumor area was measured twice weekly with a caliper gage until 28 days after tumor inoculation, with the measurements being calculated as tumor length (mm) × width (mm). Mice were considered to have “survived” when the tumor area was less than 100 mm^2^ after 28 days of tumor challenge. Each experiment had three–five mice in each group. The results were pooled from two (b) or three (d) independent experiments (*n* = 9 for the control group and *n* = 10 for the WTMCGEP group in (b); *n* = 14 for the control group, *n* = 13 for the WTMCGEP group, *n* = 6 for the control + anti-CD8 group, and *n* = 10 for the WTMCGEP + anti-CD8 group in (d)). In (a) and (c), lines represent the tumor growth of each individual mouse. In (d), the log-rank test between the control and WTMCGEP groups had a *p* value of <0.002, the log-rank test between the control and control + anti-CD8 groups had a *p* value of <0.0001, the log-rank test between the WTMCGEP and WTMCGEP + anti-CD8 groups had a *p* value of <0.0001, and the log-rank test between the control + anti-CD8 and the WTMCGEP + anti-CD8 groups had a *p* value of <0.02.

**Figure 3:** WTMCGEP augments intratumoral CD8^+^ T cell activity in CD1d^−/−^ mice. CD1d^−/−^ mice fed the control or WTMCGEP diet were subcutaneously challenged with 5 × 10^4^ CT26 cells. Twenty-eight days after tumor inoculation, the recovered TILs were stained with anti-CD45, -CD3, -CD8*β*, and -CD107a. The CD107a^+^ CD8^+^ cell proportion was determined using flow cytometry. The representative flow plots are demonstrated as CD107a^+^ CD8*β*^+^ cell percentage in TILs (a). The cumulative data of two independent experiments (*n* = 9 for the control group and *n* = 7 for the WTMCGEP group) were shown in (b). The data are expressed as means ± standard deviations. ^*∗*^*p*  <  0.04 (Student's *t* test).

**Figure 4:** WTMCGEP has no effect on the CD4^+^ Foxp3^+^ Treg cell frequency in TILs. CD1d^−/−^ mice fed the control or WTMCGEP diet were subcutaneously challenged with 5 × 10^4^ CT26 cells. Twenty-eight days after tumor inoculation, the recovered TILs were stained with anti-CD45, -CD3, -CD4, and -Foxp3. The CD4^+^ Foxp3^+^ cell proportion was determined using flow cytometry. The representative flow plots are demonstrated as CD4^+^ Foxp3^+^ cell percentage in TILs (a). We used three–five mice for each group to perform three independent experiments and pooled the results (b). Each symbol indicates one data point. The data are expressed as means ± standard deviations.

**Figure 5:** WTMCGEP reduces the proportion of both intratumoral and splenic PMN-MDSCs in CD1d^−/−^ mice. CD1d^−/−^ or WT mice fed the control or WTMCGEP diet were subcutaneously challenged with 5 × 10^4^ CT26 cells. Twenty-eight days after tumor inoculation, intratumoral and splenic leukocytes were isolated from these mice and flow cytometry was performed for detecting and measuring Ly6G^+^ Ly6C^lo^ PMN-MDSCs and Ly6G^−^ Ly6C^hi^M-MDSCs. (a), (c), (e), and (g) show representative flow data. The presented dot plots were gated on the CD45^+^ CD11b^+^ population. (b, d) show the pooled results from three independent experiments. (f, h) show the pooled results from two independent experiments. Three–five mice per group were used for each experiment. Each symbol indicates one data point. Data are expressed as means ± standard deviations. The Mann–Whitney *U*-test between the control and WTMCGEP groups in CD1d^−/−^ TILs (b left) showed a *p* value of <0.05. Student's *t* test between the control and WTMCGEP groups in CD1d^−/−^ spleens (d left) showed a *p* value of <0.04.

**Table 1:** Composition of WTMCGEP.

Crude drug	Botanical origin	Ratio (g)
*Wisteria floribunda*	Tree of *Wisteria floribunda* (Willd.) DC.	1.83
*Trapae fructus*	Fruit of *Trapa japonica* Flerow	1.83
*Myristica fragrans*	Seed of *Myristica fragrans* Houttuyn., family Myristicaceae	1.83
*Coicis semen*	Seed without husk of *Coix lachrymajobi* L. var. ma-yuen (Roman.) Stapf, family Gramineae	3.66
*Ganoderma lucidum*	Fruit body of *Ganoderma lucidum* Karst.	3.66
*Elfvingia applanata*	Fruit body of *Elfvingia applanata* Karst.	1.83
*Punica granatum*	Pericarp of *Punica granatum* L., family Punicaceae	1.83

4.5 g of WTMCGEP extract granules contains 1.5 g of a dried extract of the aforementioned mixed crude drugs. Inactive ingredient is the Japanese pharmacopeia corn starch.

## Data Availability

All data generated or analyzed during this study are included in this published article.

## Abbreviations

WTMCGEP: *Wisteria floribunda*, *Trapae fructus*, *Myristica fragrans*, *Coicis semen*, *Ganoderma lucidum*, *Elfvingia applanata*, and *Punica granatum*
Treg: Regulatory T cells
MDSCs: Myeloid-derived suppressor cells
PMN-MDSCs: Polymorphonuclear MDSCs
M-MDSCs: Monocytic MDSCs
TILs: Tumor-infiltrating lymphocytes.
